The article "Effect of Cardiac Rehabilitation Therapy Combined with WeChat Platform Education on Patients with Unstable Angina Pectoris after PCI" was published in 2022. Journal: J Healthc Eng.

# Effect of Cardiac Rehabilitation Therapy Combined with WeChat Platform Education on Patients with Unstable Angina Pectoris after PCI

**DOI:** 10.1155/2022/7253631

**Published:** 2022-03-07

**Authors:** Bin Wang, Jinsong Li, Yanling Hong, Yibin Gao, Mao Tian, Qiang Lin, Jiawei Wang, Yu Wang, Xiang Li

**Affiliations:** ^1^Department of Cardiology, Luzhou People's Hospital, Luzhou 646000, Sichuan, China; ^2^Department of Electrocardiogram, Luzhou People's Hospital, Luzhou 646000, Sichuan, China

## Abstract

**Objective:**

The aim of this study is to explore the effect of cardiac rehabilitation therapy combined with WeChat platform education on patients with unstable angina pectoris (UAP) after percutaneous coronary intervention (PCI).

**Methods:**

Eighty-eight UAP patients undergoing PCI in our hospital from June 2018 to June 2021 were chosen as the study subjects and were grouped according to the intervention methods. Specifically, patients receiving routine treatment only were included as the control group (CG) and those receiving cardiac rehabilitation therapy combined with WeChat platform education based on the routine treatment were included as the study group (SG), with 44 cases in each group. The clinical efficacy was compared between the two groups after intervention.

**Results:**

Compared with CG, SG achieved notably better biochemical indexes of TC, TG, FBG, FIB, LDL-c, and HDL-c after 12 months of intervention (*P* < 0.05), lower systolic pressure (SBP), and diastolic pressure (DBP) after intervention (*P* < 0.05), and higher scores of limited mobility, anginal stability, anginal frequency, subjective perception, treatment satisfaction, and total SAQ after 12 months of intervention (*P* < 0.05). The LVEF levels of both groups increased after intervention (*P* < 0.05), and the LVEF level was higher in SG than in CG (*P* < 0.05). The incidence of adverse cardiac events such as heart failure, ventricular arrhythmia, and sudden cardiac death was slightly higher in CG than in SG within 12 months of intervention, with no statistical difference (*P* > 0.05). The UAP recurrence rate and incidence of myocardial infarction in CG were obviously higher than those in SG (*P* < 0.05).

**Conclusion:**

Cardiac rehabilitation therapy combined with WeChat platform education intervention measures for UAP patients after PCI can effectively control the biochemical indexes such as blood lipid and blood glucose, improve the cardiac function, stabilize the disease condition, lower the recurrence rate, and reduce the incidence of other cardiac adverse events.

## 1. Introduction

With the changes of people's lifestyle and the speeding up of aging, coronary heart disease (CHD) has become the primary cause of death at home and abroad. Currently, percutaneous coronary intervention (PCI), the preferred emergency intervention treatment of CHD, mainly completes the mechanical support of the stenosis coronary artery through stent implantation, which can effectively improve the clinical symptoms and reduce the mortality in the acute stage. However, the risk of coronary restenosis or bleeding in patients after PCI affects the rehabilitation process and quality of life after intervention [1–4]. Cardiac function is the basis to ensure the efficacy of patients and good cardiac function can improve patients' tolerance to adverse factors, so effective cardiac rehabilitation therapy after PCI is particularly important for such patients. Relevant studies [5–7] have demonstrated that cardiac rehabilitation therapy can delay the development of atherosclerosis, even reverse the formation of plaques, and prevent arterial stenosis or blockage caused by thrombosis. Therefore, cardiac rehabilitation therapy was included in our hospital for patients with unstable angina (UAP) after PCI to accelerate their recovery of cardiac function. In addition, a clinical study [8, 9] has found that many risk factors affect CHD, including not only traditional factors such as age, hypertension, diabetes, dyslipidemia, and unhealthy diet but also new risk factors such as sleep apnea, abnormal high-sensitivity C-reactive protein (hsCRP), hypertriglyceridemia, and homocysteinemia. In order to improve the curative effect of PCI and reduce the influence of the above risk factors on UAP patients, intervention of patients was strengthened in our hospital through the WeChat education platform to achieve the effect of continuous nursing. Few studies have been found in terms of the effect of cardiac rehabilitation therapy combined with WeChat platform education on UAP patients after PCI. Therefore, 88 patients were included in our hospital to carry out retrospective analysis and investigate the efficacy of the joint intervention, aiming to provide reference for clinical practice.

The article "Effect of Cardiac Rehabilitation Therapy Combined with WeChat Platform Education on Patients with Unstable Angina Pectoris after PCI" was published in 2022. Journal: J Healthc Eng.

## 2. Study Protocol

### 2.1. Case Screening

The inclusion criteria were formulated according to the objectives of this study: (1) the patients were diagnosed with UAP after coronary angiography; (2) the patients underwent PCI for the first time; (3) the patients had no reperfusion arrhythmia (arrhythmia due to reperfusion after myocardial recovery) and they were hemodynamically stable after PCI; (4) the patients had no visual, hearing, or cognitive impairment; and (5) the patients and family members were informed of this study and voluntarily signed the informed consent.

Exclusion criteria: (1) those with severe myocarditis, valvular diseases, cardiomyopathy or arrhythmia; (2) those with extremely unstable disease conditions; (3) those with cardiac insufficiency (NYHA class IV); (4) those with left ventricular ejection fraction (LVEF) below 30%; (5) those with cerebrovascular diseases, pulmonary diseases, abnormal liver and kidney function, malignancy, immune system diseases, or severe diseases of limb activity; and (6) those with the installment of a pacemaker cardiac pacemaker.

Eighty-eight UAP patients undergoing PCI in our hospital from June 2018 to June 2021 were chosen as the study subjects according to the above screening criteria.

### 2.2. Grouping

The 88 patients were grouped according to the intervention methods. Specifically, patients receiving routine treatment only were included as the control group (CG) and those receiving cardiac rehabilitation therapy combined with WeChat platform education based on the routine treatment were included as the study group (SG), with 44 cases in each group. In line with the Declaration of Helsinki (as revised in 2013) [10], the study was approved by the hospital ethics committee.

### 2.3. Intervention Methods

Routine treatment. The intervention was implemented for patients with a stable condition at one week after PCI, mainly including preliminary clinical assessment, second-level prevention drugs for CHD, and health education. In addition, 24-hour ECG monitoring was performed and oxygen inhalation was provided for patients with dyspnea. Besides, repeated detection of myocardial necrosis markers was carried out if necessary [3, 11].

Cardiac rehabilitation therapy. (1) The therapy included 5–10 min of warm-up exercise and 20–30 min of cardiac rehabilitation exercise. Rehabilitation the exercise contained aerobic and resistance exercises. Aerobic exercise was achieved by running or jogging on treadmills and cycling, requiring real-time ECG monitoring during exercise and was supplemented with flexibility and balance training when necessary. Then, 5–10 min of relaxation exercise was carried out at the end of the rehabilitation. (2) The exercise intensity was set according to the target heart rate (60–80% of the maximum heart rate after age standardization) [12, 13]. (3) After discharge, patients could choose one or several types of aerobic exercise such as walking, jogging, cycling, Taiji, swimming, and dancing, with the same exercise intensity and time as those in the hospital, and 3–5 times a week. (4) The patients were assessed every 2 weeks in the physicians' outpatient clinics, and the exercise programs were adjusted if necessary.

WeChat platform education. The health education was carried out on the family members of patients through the WeChat platform, specifically as follows. The primary nurses established a WeChat group and added the head nurse, the department director, medical staff, UAP patients undergoing PCI in the department, and their families in the group. The group was named as *health education group (after PCI).* The main tasks of the primary nurses were as follows. (1) Electronic records were established for all patients, including basic information and changes of the condition. The records of the patients were screened every week, and those who needed to be reviewed were informed in the WeChat group. After review, the results were uploaded to the WeChat group. The nursing staff also organized the results into electronic records and registered them well. (2) Patients were asked every Tuesday to upload the photos of their blood glucose and blood pressure in the last week to the WeChat group for registration. (3) Patients and their families were instructed to feel and observe the symptoms of angina pectoris such as chest distress, palpitation and chest pain, and their families were instructed to observe whether patients had symptoms of heart failure such as panting, cough, and swelling of lower limbs. (4) The CHD-related health knowledge was regularly updated on the WeChat platform, mainly including the prevention of hypertension, diabetes and angina pectoris, CHD risk factors, dietary guidance, lifestyle advice, PCI-related knowledge, the influence of adverse factors on UAP after PCI, and the impact of bad lifestyle on patients. The patients and family members were also informed of the taboo behaviors, and the families were encouraged to supervise the patients [14]. (5) The patients could carry out one-to-one consultations from 8.30 to 10.30 a. *m*. every day within the group and raised questions about daily life and diseases, which would be answered by the specialized medical staff. (6) The family members were taught first aid general knowledge such as how to correctly perform cardiopulmonary resuscitation and dialing 120 in case of emergency.

The article "Effect of Cardiac Rehabilitation Therapy Combined with WeChat Platform Education on Patients with Unstable Angina Pectoris after PCI" was published in 2022. Journal: J Healthc Eng.

### 2.4. Observation Indexes

The age, gender, smoking, drinking, diabetes, hyperlipidemia, hypertension, NYHA classification, and the number of diseased vessels were statistically analyzed. The biochemical indexes of both groups after 12 months of intervention were analyzed, including total cholesterol (TC), triglyceride (TG), fasting blood glucose (FBG), fibrinogen (FIB), low density lipoprotein cholesterol (LDL-c), and high density lipoprotein cholesterol (HDL-c). The blood pressure levels were also analyzed after intervention, namely, systolic pressure (SBP) and diastolic pressure (DBP).

The *Seattle Angina Questionnaire (SAQ)* [15] was adopted for evaluating the recovery of angina pectoris, mainly including limited mobility, anginal stability, anginal frequency, subjective perception, and treatment satisfaction, with each scoring 100 points. Higher scores demonstrated better physical condition of the patients. The LVEF levels before and after intervention were measured by color Doppler ultrasound to evaluate the cardiac function. The occurrence of adverse cardiac events such as recurrent UAP, myocardial infarction, heart failure, ventricular arrhythmia, and sudden cardiac death within 12 months of intervention were analyzed.

### 2.5. Statistical Treatment

The data were calculated by software SPSS22.0, and graphed by software GraphPad Prism 7 (GraphPad Software, San Diego, USA). The data included are enumeration and measurement data, which were expressed as [*n* (%)] and ($\bar{x}$ ± *s*), and tested by *X*^2^ and *t*-test. When *P* < 0.05, the differences were statistically significant.

## 3. Results

### 3.1. General Information

Table 1 presents no notable differences in general data such as age, gender, smoking, drinking, diabetes, hyperlipidemia, hypertension, NYHA classification, and the number of diseased vessels between the two groups (*P* < 0.05).

### 3.2. Biochemical Indexes

As shown in Table 2, after 12 months of intervention, the biochemical indexes such as TC, TG, FBG, FIB, LDL-C, and HDL-C were remarkably better in the SG than in the CG (*P* < 0.05).

### 3.3. Blood Pressure Levels

As presented in Figure 1, SBP and DBP after intervention in the SG were obviously lower compared with the CG (*P* < 0.05).

### 3.4. Angina Pectoris

After 12 months of intervention, SG had higher scores of limited mobility, anginal stability, anginal frequency, subjective perception, treatment satisfaction, and total SAQ compared with CG (*P* < 0.05), see Figure 2.

### 3.5. Cardiac Function

The LVEF levels of both groups increased after intervention (*P* < 0.05), and the LVEF level was higher in the SG than in the CG (*P* < 0.05), as presented in Table 3.

### 3.6. Incidence of Adverse Cardiac Events

The incidence of adverse cardiac events such as heart failure, ventricular arrhythmia, and sudden cardiac death was slightly higher in the CG than in the SG within 12 months of intervention, with no statistical difference (*P* > 0.05). The UAP recurrence rate and incidence of myocardial infarction in the CG were obviously higher than those in the SG (*P* < 0.05), see Table 4.

## 4. Discussion

In 2007, the World Health Organization (WHO) issued the *Guidelines for Evaluation and Management of Cardiovascular Risk Factors*, which clearly pointed out that the incidence and mortality of cardiovascular diseases were closely related to individual exercise regardless of gender and age [16–19]. At present, plenty of relevant studies at home and abroad have shown that cardiac rehabilitation therapy is one of the most important treatment methods in second-level prevention of CHD after PCI. European Society of Cardiology, American Heart Association, and American College of Cardiology have included the therapy as the level I recommendation in the CHD treatment guidelines [20–23]. Cardiac rehabilitation therapy is an interdisciplinary and comprehensive rehabilitation system, including cardiovasology, kinematics, rehabilitation, nutrition, and psychology. Effective cardiac rehabilitation measures cannot only reduce the mortality of CHD patients after PCI but also reduce the readmission rate and the incidence of adverse cardiac events. However, clinical investigation shows that the promotion and application of cardiac rehabilitation therapy are still hindered by low clinical participation and high dropout rates of patients. In addition, with the continuous development of the smart medical industry, health education based on the WeChat platform has gradually been promoted. It mainly strengthens the intervention of patients and their families with the help of modern mobile terminals. On the one hand, it improves the patients' disease cognition and compliance behaviors from two aspects of the psychological state and behavioral constraints. On the other hand, it enriches the forms of communication between doctors and patients, greatly improves the efficiency of clinical intervention, and makes great progress in health education.

The article "Effect of Cardiac Rehabilitation Therapy Combined with WeChat Platform Education on Patients with Unstable Angina Pectoris after PCI" was published in 2022. Journal: J Healthc Eng.

Unstable angina pectoris (UAP), a kind of acute coronary syndrome, is a clinical state between stable angina pectoris and acute myocardial infarction, which is closely related to factors such as age, gender, dyslipidemia, hypertension, diabetes, and smoking. Even after PCI, patients still face a high risk of recurrence. If patients have large areas of myocardial infarction, the condition is dangerous and even life-threatening. In recent years, based on the clinical nursing needs of such patients, our hospital has implemented cardiac rehabilitation therapy combined with WeChat platform education and found that the recurrence rate of angina pectoris tends to decrease, but there are few related studies on their combination. Based on this, clinical intervention was performed on some UAP patients after PCI in our hospital. The results showed that compared with the CG, the SG achieved notably better biochemical indexes of TC, TG, FBG, FIB, LDL-c, and HDL-c after 12 months of intervention (*P* < 0.05), and lower SBP and DBP after intervention (*P* < 0.05). These results were similar to the study of Heber [24], further confirming that cardiac rehabilitation therapy combined with WeChat platform education can effectively control and improve the blood pressure, blood lipid, and blood glucose levels of patients. In addition, after 12 months of intervention, the SG had higher scores of limited mobility, anginal stability, anginal frequency, subjective perception, treatment satisfaction, and total SAQ compared with the CG (*P* < 0.05). The LVEF levels of both groups increased after intervention (*P* < 0.05), and the LVEF level was higher in the SG than in the CG (*P* < 0.05). The incidence of adverse cardiac events such as heart failure, ventricular arrhythmia, and sudden cardiac death was slightly higher in the CG than in the SG within 12 months of intervention, with no statistical difference (*P* > 0.05). The UAP recurrence rate and incidence of myocardial infarction in the CG were obviously higher than those in the SG (*P* < 0.05). The above results suggested that cardiac rehabilitation therapy combined with WeChat platform education better controlled the condition of UAP patients, enhanced the body activity, reduced anginal frequency and improved subjective feelings. The LVEF levels of patients demonstrated the combined intervention also improved the heart function of patients and reduced the probability of adverse cardiac events.

The article "Effect of Cardiac Rehabilitation Therapy Combined with WeChat Platform Education on Patients with Unstable Angina Pectoris after PCI" was published in 2022. Journal: J Healthc Eng.

PCI is an important treatment for UAP patients in the acute stage. However, patients still face long-term and arduous rehabilitation tasks after the stable condition, mainly including the improvement of body endurance and cardiac function, and the requirement of healthy behaviors. Cardiac rehabilitation therapy can increase blood flow and oxygen consumption of skeletal muscles, expand peripheral capillaries, reduce resistance, and thus reduce blood pressure. In addition, cardiac rehabilitation therapy cannot only reduce the levels of TC, TG, and LDL-c in blood, which are risk factors for the formation of atherosclerotic plaques, but also increase the antiatherosclerotic HDL-c level. The mechanism may be that cardiac rehabilitation therapy increases the activity of lipoprotein lipase, accelerates the TG decomposition, and increases HDL-c by LDL-c cleavage. Cardiac rehabilitation therapy can also increase the content of glucose transporters in skeletal muscle cells and promote the uptake and utilization of blood glucose in the body, thus playing a hypoglycemic effect. Therefore, cardiac rehabilitation therapy can lay a good foundation for antiatherosclerosis, but the good treatment effect may not last for a long time if the intervention of a healthy diet and lifestyle is not strengthened. Supported by the Internet, WeChat platform education strengthens the intervention of patients after PCI in the form of text, voice, pictures and videos, popularizes health education through WeChat to enhance patients' understanding of the disease, and timely deals with the condition changes to reduce the incidence of adverse cardiac events. By advocating a healthy lifestyle and eating habits, the patients' indicators such as blood glucose, blood pressure, and blood lipids are controlled well to create a good environment for the recovery of cardiac function. WeChat platform education intervention and cardiac rehabilitation therapy cooperate with and complement each other. This study also has some inadequacies, such as small sample size, inadequate forms of cardiac rehabilitation training, and the incomplete WeChat education platform. Therefore, it is also necessary to expand the sample size, enrich the forms of cardiac rehabilitation, improve the WeChat education platform, and establish a long-term and effective follow-up mechanism.

The article "Effect of Cardiac Rehabilitation Therapy Combined with WeChat Platform Education on Patients with Unstable Angina Pectoris after PCI" was published in 2022. Journal: J Healthc Eng.

In conclusion, cardiac rehabilitation therapy combined with WeChat platform education intervention measures for UAP patients after PCI can effectively control the biochemical indexes such as blood lipid and blood glucose, improve the cardiac function, stabilize the disease condition, lower the recurrence rate, and reduce the incidence of other cardiac adverse events.

## Figures and Tables

**Figure 1:** Statistics of blood pressure levels after intervention ($\bar{x}$ ± *s*). Note: The abscissa represented SBP and DBP, and the ordinate represented the blood pressure (mmHg). The SBP and DBP after intervention were (131.75 ± 9.06) and (83.16 ± 9.11) in the CG, and (124.65 ± 8.14) and (76.10 ± 8.24) in SG. ^*∗*^indicates a notable difference in SBP between the two groups (*t* = 3.867, *P* < 0.001). ^*∗∗*^indicates a notable difference in DBP between the two groups (*t* = 3.812, *P* < 0.001).

**Figure 2:** Statistics of SAQ scores after 12 months of intervention ($\bar{x}$ ± *s*). Note: The abscissa represented the evaluation dimensions and the ordinate represented the score (points). In the CG, the scores of limited mobility, anginal stability, anginal frequency, subjective perception, treatment satisfaction, and total SAQ were (91.84 ± 2.11), (74.85 ± 3.52), (74.86 ± 2.60), (75.14 ± 2.59), (80.01 ± 5.20), and (77.86 ± 2.40). In the SG, the scores of limited mobility, anginal stability, anginal frequency, subjective perception, treatment satisfaction, and total SAQ were (93.55 ± 2.04), (79.88 ± 3.45), (79.56 ± 2.47), (80.05 ± 2.37), (89.04 ± 5.14), and (84.12 ± 2.19). ^∗^from left to right indicates notable differences in the scores of limited mobility, anginal stability, anginal frequency, subjective perception, treatment satisfaction, and total SAQ between the two groups (*t* = 3.865, 6.769, 8.693, 9.277, 8.192 and 12.781; *P* < 0.001).

The article "Effect of Cardiac Rehabilitation Therapy Combined with WeChat Platform Education on Patients with Unstable Angina Pectoris after PCI" was published in 2022. Journal: J Healthc Eng.

**Table 1:** Comparison of general data (*n* = 44).

Observation indexes	CG	SG	X^2^/*t*	*P*
Age (years old)	55.41 ± 7.50	56.12 ± 7.62	0.440	0.661
Gender (male/Female)	35/9	36/8	0.073	0.787
Smoking	24 (54.55)	22 (50)	0.182	0.669
Drinking	21 (47.73)	19 (43.18)	0.183	0.669
Diabetes	5 (11.36)	6 (13.64)	0.104	0.747
Hyperlipidemia	18 (40.91)	17 (38.64)	0.047	0.828
Hypertension	27 (61.36)	25 (56.82)	0.188	0.665
NYHA classification				
I	12 (27.27)	15 (34.09)	0.481	0.488
II	27 (61.36)	25 (56.82)	0.188	0.665
III	5 (11.36)	4 (9.09)	0.124	0.725
Number of diseased vessels				
Single	25 (56.82)	26 (59.09)	0.047	0.829
Double	13 (29.55)	14 (31.82)	0.053	0.817
Triple	6 (13.64)	4 (9.09)	0.451	0.502

**Table 2:** Statistics of biochemical indexes after 12 months of intervention ($\bar{x}$ ± *s*).

Biochemical indexes	CG	SG	*t*	*P*
TC (mmol/L)	6.09 ± 0.20	5.45 ± 0.23	13.928	<0.001
TG (mmol/L)	1.88 ± 0.16	1.66 ± 0.21	5.032	<0.001
FBG (mmol/L)	6.83 ± 0.34	6.25 ± 0.27	8.861	<0.001
FIB (g/L)	4.22 ± 0.28	3.71 ± 0.19	9.998	<0.001
LDL-c (mmol/L)	3.19 ± 0.35	2.76 ± 0.28	6.364	<0.001
HDL-c (mmol/L)	1.15 ± 0.10	1.45 ± 0.18	9.664	<0.001

**Table 3:** Statistics of LVEF levels after intervention ($\bar{x}$ ± *s*).

Group	*n*	Before intervention	After intervention
CG	44	51.08 ± 4.71	57.88 ± 5.04^*∗*^
SG	44	50.93 ± 4.85	63.10 ± 4.25^*∗*^
*t*		0.147	5.252
*P*		0.883	<0.001

^*∗*^indicates an obvious difference in the LVEF levels before and after intervention within the same group (*P* < 0.05).

**Table 4:** Statistics of incidence of adverse cardiac events after intervention (‾*x* ± *s*).

Group	Recurrence UAP	Myocardial infarction	Heart failure	Ventricular arrhythmia	Sudden cardiac death
CG	8 (18.18)	6 (13.64)	4 (9.09)	3 (6.82)	1 (2.27)
SG	2 (4.55)	1 (2.27)	1 (2.27)	1 (2.27)	0 (0)
*X* ^*2*^	4.062	3.880	1.908	1.048	1.012
*P*	0.044	0.049	0.167	0.306	0.315

## Data Availability

The data used to support the findings of this study are available on reasonable request from the corresponding author.
